The article "Application of Artificial Intelligence within Virtual Reality for Production of Digital Media Art" was published in 2022. Journal: Comput Intell Neurosci.

# Application of Artificial Intelligence within Virtual Reality for Production of Digital Media Art

**DOI:** 10.1155/2022/3781750

**Published:** 2022-08-10

**Authors:** Yunxuan Wu

**Affiliations:** ^1^College of Culture and Communication, Liming Vocational University, Quanzhou, Fujian 362000, China; ^2^Graduate University of Mongolia, Ulaanbaatar 14192, Mongolia

## Abstract

As technology changes, virtual reality generates realistic images through computer graphics and provides users with an immersive experience through various interactive means. In the context of digitalization, the application of VR for digital media art creation becomes a normalized method. Today's digital media art creation is closely related to vigorous technological innovation behind it, so the influence of modern technology is inevitable. Virtual reality and artificial intelligence have gradually become the main technical means in line with the development aim for digital media art creation. This work proposes an art object detection method AODNET in virtual reality digital media art creation with AI. Aiming at the particularity of object detection in this direction, an art object detection strategy based on residual network and clustering idea is proposed. First of all, it uses ResNet50 as backbone, which deepens network depth and improves the model feature extraction ability. Second, it uses the K-means++ algorithm to perform clustering statistics on the size of the real annotated boxes in the dataset to obtain appropriate hyperparameters for preset candidate boxes, which enhances the tolerance of the algorithm to the target size. Third, it replaces the ROI pooling algorithm with ROI align to eliminate the error caused by the quantization operation on the characteristics of the candidate region. Fourth, to reduce the missed detection rate of overlapping targets, soft-NMS algorithm is used instead of the NMS algorithm to post-process the candidate boxes. Finally, this work conducts extensive experiments to verify the superiority of AODNET for object detection in virtual reality digital media art creation.

## 1. Introduction

VR technology is to create virtual environment through the application of computer operation and image technology. This virtual environment is a dynamic and perceptible simulation environment, in which users can perceive and obtain relevant information through physical senses. Since the simulation environment constructed by VR technology adopts 3D modeling technology, the rendered scene is relatively realistic. Coupled with the application of some other technologies, users can perceive information in the VR environment through vision, hearing, touch, and even smell and taste, so that users are immersed in it, and the transmission of information becomes more direct and specific. Artificial intelligence technology refers to a technology that imitates the consciousness and thinking cognition of the human brain through computer technology and on the basis of big data. As an interdisciplinary frontier discipline, artificial intelligence covers a series of disciplines such as mathematics, computer science, psychology, statistics, and biology and integrates knowledge. This enables it to perform simple self-learning and achieve intelligence. At present, although artificial intelligence technology has not been fully applied to life, the prototype of aAI applications has been seen in many industries. It will become the main technical support for various industries in the future [1–5].

The article "Application of Artificial Intelligence within Virtual Reality for Production of Digital Media Art" was published in 2022. Journal: Comput Intell Neurosci.

The traditional approach of creating digital media art is straightforward, but it also necessitates a high level of imagination and perception on the part of the artist. Because of this, creating a work of digital media art requires a significant investment of time, energy, and materials. The advent and development of AI and VR technologies, however, have given rise to new idea for digital media art in the current social context. To a certain extent, this lessens the difficulty of digital media art creation and improves producers' job efficiency and their work quality. Work in diverse forms and unique creation processes are continually appearing as a result of involvement of virtual reality in digital media art. As the VR and AI have grown, it has range of digital media art forms and content available [6–10].

With VR, the makers of digital media art can not only experience a virtual world, but they can also keep their biological perceptions as well. As a result, it might provide a sense of immersion, which is extremely advantageous to the creative process of the creator. To provide a pleasant experience from start to finish, virtual reality's artificial intelligence may adapt to the preferences of the user. To the designers of digital media art, virtual reality technology can provide a unique experience because it is a front-end technology that includes a wide range of functionalities. It is possible to create a more lifelike virtual reality experience by utilizing artificial intelligence in conjunction with the enhanced three-dimensional perception provided by human vision. The artificial intelligence of VR technology can also help digital media artists gather a large amount of data, giving them a better understanding of how their methods of information transmission differ from others. VR can be used to create three-dimensional sensation of immersion in the virtual environment by digital media artists. Because of the great capabilities of virtual reality's artificial intelligence application, it is possible to immerse oneself in the virtual world and improve one's effectiveness and breadth in receiving information from it. When seeing digital media artworks in the past, people relied solely on view. All the senses can be activated when appreciating these works under influence of science, resulting in greater realism and a more authentic experience. With the help of artificial intelligence, virtual reality may be used to its greatest potential, allowing users to gain a deeper understanding of creators and goals for their works. VR's artificial intelligence challenges and expands the creative possibilities of digital media artists, according to their perspective. Because virtual reality art is created using artificial intelligence and relies on digital media, it is safe to assume that digital media has played a significant role in shaping its organizational structure and aesthetic attributes. Although digital media art is still a form of art, its unique characteristics need a shift in the way people view and appreciate it [11–15].

The article "Application of Artificial Intelligence within Virtual Reality for Production of Digital Media Art" was published in 2022. Journal: Comput Intell Neurosci.

Aiming at the particularity of object detection in digital media art creation of virtual reality, this work proposes an art object detection algorithm based on residual network and clustering idea. First of all, it uses ResNet50 as the feature extraction network, which deepens the network depth and improves the model feature extraction ability. Second, it uses the K-means++ algorithm to perform clustering statistics on the size of the real annotated boxes in the dataset to obtain appropriate hyperparameters for preset candidate boxes, which enhances the tolerance of the algorithm to the target size. Third, it replaces the ROI pooling algorithm with ROI align to eliminate the error caused by the quantization operation on the characteristics of the candidate region. Fourth, to reduce missed detection rate of overlapping targets, soft-NMS algorithm is used instead of the NMS algorithm to post-process the candidate boxes. Finally, this work conducts extensive experiments to verify the superiority of AODNET for object detection in virtual reality digital media art creation.

## 2. Related Work

Reference [16] analyzed some basic characteristics and development of virtual reality technology and made a general analysis of future applications. However, the writing time of the article was relatively early, the analysis process was brief, and the examples cited in the article were also the artist's own vision, and at that time, there was no suitable case to prove it. Literature [17] not only systematically introduced the technology, application, history, and development issues involved in VR virtual technology but also introduced how to use virtual technology in art. This was a large-scale introduction to some big concepts, and the author also explained it from the perspective of a virtual reality technology researcher. Literature [18] made clear expectations for the combination of virtual reality and art and analyzed several important factors for the combination of the two: the development of art in the computer age, the subjective exploration of artists, and the needs of audiences. Literature [19] compared VR technology with the current Internet and genetic engineering. At the same time, it introduced many artists who used virtual reality technology as a means to create and also introduced various types of virtual art. Literature [20] roughly talked about the impact of virtual reality technology on artistic creation, teaching, and the application of installation art, conceptual art, and urban public art. It briefly introduced that virtual reality technology would be used in this area, but there was no specific and in-depth analysis, and the research was not detailed and rigorous enough. Literature [21] proposed that with the development of virtual reality technology, new conditions and requirements were provided for the application of art in teaching, and a lot of practice had proved that virtual reality technology was very effective in art teaching. An in-depth look at the existing and potential future effects of virtual reality on our daily lives may be found in the literature [22]. It considered how virtual reality could be used in a wide range of industries, as well as its creative and entertainment applications. It argued idealists' enthusiasm for computerized life that must be balanced with the need for a deeper understanding of basic reality. Reference [23] analyzed the virtual reality in the past few years, the new hardware had been entering the market, and the price was reasonable. The driving force of virtual reality was not only in the scientific community, but more and more enthusiasts were also expanding with new technologies. The situation of virtual reality in the field of commodities was becoming more and more important, and it was said that the current technology was already very powerful.

The article "Application of Artificial Intelligence within Virtual Reality for Production of Digital Media Art" was published in 2022. Journal: Comput Intell Neurosci.

Reference [24] proposed R-CNN, a classic work that applied deep learning technology to target detection. Its main steps were divided into two parts: target candidate region generation and accurate classification and regression, which were called two-stage target detection. Reference [25] proposed the SPPNet algorithm, which used full-image convolution as feature extraction, and proposed a spatial pyramid pooling network structure. Reference [26] proposed Fast-RCNN, performed ROI pooling on the feature map to obtain the sampled feature map, and used the multitask loss to realize the end-to-end network training process. Reference [27] proposed faster R-CNN, which uses RPN to realize target candidate region screening with a convolutional neural network and proposed to encode and assign targets in the way of anchor. It defined the network position output as the relative relationship with the anchor box, so that the whole process task was completed by the neural network structure. Reference [28] proposed feature FPN, which developed a top-down horizontal connection structure to form a feature pyramid for the problem that the low resolution of deep networks was not conducive to accurate regression. Reference [29] pioneered the use of a single-stage network structure to complete the target detection task and proposed the YOLO algorithm. It did not use the RPN structure to perform coarse-grained estimation of the target existence area, but directly regarded target detection as a regression problem and predicted that the target position represented by each pixel position on the feature map was in the target category. Reference [30] assigned different scale targets to feature maps of different resolutions as output, which improved the detection ability of the algorithm for small-scale targets. Reference [31] analyzed the reasons why the performance of the single-stage detection lagged behind the two-stage detection algorithm. The conclusion was that the single-stage detection algorithm had a process similar to dense sampling, which led to extremely serious sample imbalance in the process of positive and negative sample assignment. Therefore, the focal loss was proposed, which enabled network to obtain a higher loss for the allocation of few samples and difficult samples during the training process, so as to control the bias of the algorithm. Reference [32] proposed CornerNet, which defined the object detection task as a key point regression task. It defined the supervision signal of the key point as a Gaussian patch whose variance was determined by the target scale, proposed a corner pooling structure, and assigned the network output as the heat map composed of upper left and lower right corners of bounding box as key points to be regressed. The CenterNet proposed in the literature [33] inherited the idea of key point detection, took the center position of the target as the key point to be returned, and could be extended to tasks such as monocular 3D detection and pose estimation. This kind of target detection algorithm based on Gaussian spot detection as a key point used the positive sample representation of the target at the maximum value position in the heat map, thereby replacing the non-NMS process in other detection algorithms.

The article "Application of Artificial Intelligence within Virtual Reality for Production of Digital Media Art" was published in 2022. Journal: Comput Intell Neurosci.

## 3. Method

Aiming at the particularity of object detection in digital media art creation of VR, this work proposes an art object detection algorithm AODNET based on residual network and clustering idea. First of all, it uses ResNet50 as the feature extraction network, which deepens the network depth and improves the model feature extraction ability. Second, it uses the K-means++ algorithm to perform clustering statistics on the size of the real annotated boxes in the dataset to obtain appropriate hyperparameters for preset candidate boxes, which enhances the tolerance of the algorithm to the target size. Third, it replaces the ROI pooling algorithm with ROI align to eliminate the error caused by the quantization operation on the characteristics of the candidate region. Fourth, to reduce the missed detection rate of overlapping targets, soft-NMS algorithm is used instead of the NMS algorithm to post-process the candidate boxes.

### 3.1. Convolutional Neural Network

CNN is a kind of feedforward network whose function is similar to that of multilayer perceptron. Convolutional neural networks are mainly composed of multilayer convolutional layers and the convolution kernels they contain. To ensure nonlinear transformation between convolutional layers and efficient computing process, its network components also include activation layers and pooling layers. Finally, the final output is obtained through the fully connected layer, the loss value is calculated in the objective function, and the partial derivative of the objective function to each layer is calculated through backpropagation, to update the weight parameters of the network, so that the network can learn from the data.

The convolutional layer is composed of multiple convolution kernels and is the basic structure of CNN. The main function is extracting local features. The essence of convolution is many multidimensional matrices responsible for saving the parameters learned by the network. Each convolution kernel has the characteristics of local receptive field and weight sharing for the input image, which can reduce the computational complexity and parameters compared with traditional ANN. In a convolutional neural network, the convolution kernel of each layer is only connected to some of the convolution kernels of the previous layer, the low-level convolution kernel is responsible for extracting local features, and a high-level convolution kernel is responsible for integrating feature information to obtain global feature map. Compared with fully connected layer, the partial connection method can better alleviate the problem of overfitting, reduce parameters, and speed up the convergence speed of network. The weight-sharing feature of the convolution kernel is that the convolution kernel shares the same set of parameter operations in all regions of the input feature map. However, since the convolution kernel extracts the local features of the input image, each convolution kernel can only extract fixed features. Therefore, by increasing convolution kernels, image attributes that can be extracted by the convolution layer can be increased. Convolutional layers of different depths can extract different features, and feature maps extracted by low-level convolutions learn local features due to the small receptive field. A high-level feature map is composed of low-level feature maps, so the convolution kernel can extract more complex and comprehensive features. The convolution is calculated as follows:

(1) $$\begin{array}{c} \text{Conv}\left(x\right)=\sum_{i}w_{i}x_{i}, \end{array}$$

where *w* is weight and *x* is feature.

The article "Application of Artificial Intelligence within Virtual Reality for Production of Digital Media Art" was published in 2022. Journal: Comput Intell Neurosci.

The pooling layer is usually connected after a single or multiple convolutional layers, and its main function is to simplify the total amount of parameters and computation of the entire model by reducing feature map size. This can also increase the receptive field of convolution kernel, ensure the invariance of the network, and prevent overfitting during network training. Average pooling is to calculate the average value, and max pooling selects the maximum value. Both of these operations can increase the nonlinearity of the feature and reduce the error caused by feature extraction. The error mainly comes from two aspects. Average pooling can reduce the increase in error due to the limited field size and can retain more background information of the input image. Maximum pooling can reduce the estimated value shift caused by the error of the convolution kernel parameters and can retain more texture information of the input image. The main function of global pooling is to replace the FC layer and convert the feature map into a one-dimensional feature and pass it into the classifier for classification. The fully connected layer has the disadvantage of limited input dimension. The input feature map needs to be converted and spliced into a one-dimensional vector before it can be calculated, and the number of parameters is very large. Therefore, global pooling can directly calculate a one-dimensional feature vector.

The activation layer mimics the reflex function of neurons by modeling its design after the human neural network. The classifier cannot discriminate between the abovementioned convolutional and pooling layer operations on the image because they are linear transformations. Therefore, the extracted feature map can be nonlinearly mapped through the nonlinear activation function, thereby enhancing the expressive ability of the feature. The commonly used activation functions are as follows:

(2) $$\begin{array}{c} \text{Sigmoid}\left(x\right)=\frac{1}{\left(1+e^{-x}\right)},\\ \text{Tanh}\left(x\right)=\frac{\left(e^{x}-e^{-x}\right)}{\left(e^{x}+e^{-x}\right)},\\ \text{ReLU}\left(x\right)=\max\left(0,x\right), \end{array}$$

where *x* is feature.

The article "Application of Artificial Intelligence within Virtual Reality for Production of Digital Media Art" was published in 2022. Journal: Comput Intell Neurosci.

FC layer basically corresponds to a convolutional layer of 1 × 1. The fully connected layer takes input features from the previous layer and performs a global analysis on the output features of all previous layers. Then, a nonlinear combination is performed, so it is generally used at the end of the network for classification tasks.

### 3.2. Combination of ResNet and Faster R-CNN

The shallow network can extract the simple outline information of the target, and the deep network can extract complex semantic information. However, with the deepening of the number of network layers, the model training process is difficult to converge, and classification accuracy is hard to improve. The special residual structure in ResNet subtly alleviates the problems of gradient dispersion, gradient explosion, and insignificant network performance improvement when the network depth is deepened. The idea of residual network draws on the definition of residual in statistics, and the residual is the difference between actual observed value and fitted value. Suppose one of the residual units in the residual network has to learn a mapping, but this mapping is difficult to learn directly. The residual network then transforms the original complex mapping into a simple summation operation.

Figure 1 is a schematic diagram of the residual unit. There are two branches when the feature is input into the network. One is the direct identity mapping branch without any processing. The other is the mapping branch obtained after the feature is convolutional, normalized, and activated. Then, at the confluence of the two branches, a linear superposition operation is performed on them to obtain output for the residual unit.

(3) $$\begin{array}{c} x_{l+1}=\text{ReLU}\left(x+F\left(x\right)\right), \end{array}$$

where *x* is feature and *F* is residual function.

The residual unit realizes the identity mapping of the deep network without increasing the computational cost by using a shortcut connection, which ensures the smooth transfer of the gradient and the continuous increase in the network depth. Compared with the original feature extraction layers ZF and VGG, ResNet has a deeper network layer and can extract deeper and more abstract target features. Moreover, the residual structure in ResNet is beneficial to solve the problems of gradient dispersion, gradient explosion, and insignificant network performance improvement when the network depth is deepened. In this study, ResNet50 is selected as the basic backbone. ResNet50 structure is demonstrated in Table 1.

The article "Application of Artificial Intelligence within Virtual Reality for Production of Digital Media Art" was published in 2022. Journal: Comput Intell Neurosci.

The original faster R-CNN algorithm uses VGG and ZF as the feature extraction network. If conv 1 to conv 5 of the residual network are directly combined with faster R-CNN as a new feature extraction network, although the depth is increased, model accuracy has not been effectively improved. To solve this issue, feature extraction layer is deepened and the target detection accuracy is not improved significantly, and this study adopts the networks on convolutional feature map structure (NoCs), and the specific structure is illustrated in Figure 2.

The NoCs uses conv 1 to conv 4 in ResNet50 as feature extraction layers and conv 5 and fully connected layers as the final detection subnetwork. Moving conv 5 to the detection subnetwork improves the classifier performance and thus the overall detection accuracy.

### 3.3. Cluster-Based Optimization for Preset Candidate Box

In the target detection and regression task based on a regional convolutional neural network, the degree of agreement between the size of the anchor and the real candidate box size of the target in the experimental dataset is one of the important reasons that affect the detection results. During the model training process, iterative learning will be performed according to the preset anchors, and the width and height are adjusted in time. If the size and scale of the initial proposal box of the prediction layer are properly selected, the model will soon be close to the real sample, saving training time and improving detection accuracy. The original faster R-CNN presets three sizes and three scales of boxes.

To improve the detection effect, this study uses the K-means clustering idea in the YOLO algorithm to perform clustering statistics on the real proposal boxes in the dataset and can obtain more scientific preset candidate box size and proportional hyperparameters. K-Means is a classic unsupervised learning clustering algorithm. The idea of K-means is to assign all points in the dataset to K clusters by distance division, ensuring that the distance between each sample data point and centroid of cluster to which it belongs is the closest among all cluster distances. K-Means algorithm first randomly selects K objects as the initial cluster centers according to the expected number of clusters K. Second, it calculates the distance from the remaining sample points to each cluster center and assigns it to cluster center with the smallest distance to form K clusters. Third, the average distance of all sample points is recalculated in each cluster center to the centroid. It is compared with the average distance of other sample points in the cluster, and the sample point with the smallest average distance in the cluster is selected as the new centroid. Fourth, new clusters are formed based on the new centroids, and the error sum of squares for the new clusters is recorded. Fifth, steps 2 and 3 are repeated until the end condition is reached.

The article "Application of Artificial Intelligence within Virtual Reality for Production of Digital Media Art" was published in 2022. Journal: Comput Intell Neurosci.

The K-means algorithm used in the YOLO algorithm cannot completely converge to the global optimal value due to the random determination of the initial centroid and K value. It can only converge to the local optimum and is greatly disturbed by abnormal data. Therefore, this work adopts K-means++ strategy, which improves clustering accuracy and speed by improving the method of initializing cluster centers. The biggest difference between K-means++ and K-means is the selection of initial clustering center. First, a data point is randomly selected from the dataset as the first cluster center. Second, the distance between the remaining points in dataset and existing cluster centers is calculated, and the shortest distance is selected among them. Third, the probability that each data point is utilized as the next cluster center according to (4) is calculated, and the point with the highest probability is utilized as the new cluster center. Fourth, the first to third steps are repeated until K initial cluster center points are selected, and the remaining steps are the same as the K-means algorithm.

(4) $$\begin{array}{c} p=\frac{D^{2}}{\sum D^{2}}, \end{array}$$

where *D* is distance.

The commonly used K-means++ clustering algorithm is aimed at scattered data points, and it is very appropriate to use Euclidean distance as a metric for data point classification. However, in the target detection task, the dataset to be divided is not a scattered data point, but a set of length and width values of candidate boxes. When detecting objects, the higher the overlap between the two candidate boxes, the more likely they contain the same object, and the more they should be classified into the same class. Therefore, the metric in this study does not use Euclidean distance but uses the following index to extract the size of the preset frame in the experiment.

(5) $$\begin{array}{c} d\left(\text{box},\text{centroid}\right)=1-\text{IOU}\left(\text{ox},\text{centroid}\right),\\ \text{IOU}\left(\text{box},\text{centroid}\right)=\frac{\left(S_{\text{box}}\cap S_{\text{centroid}}\right)}{\left(S_{\text{box}}\cup S_{\text{centroid}}\right)}, \end{array}$$

where box represents the real labeled box sample, centroid represents the existing cluster center, *IOU* represents the intersection ratio between the sample box and the cluster center box, *S*_box_ represents the area of sample box, and *S*_centroid_ is area of cluster center box.

The article "Application of Artificial Intelligence within Virtual Reality for Production of Digital Media Art" was published in 2022. Journal: Comput Intell Neurosci.

When the K-means++ algorithm selects a new cluster center point, the farther the distance is, the greater the probability of being selected and the greater the possibility of becoming the next cluster center, and finally, the preset cluster center is obtained.

### 3.4. ROI Align Algorithm

The ROI pooling layer undergoes two quantization operations during training. One time is to convert the coordinates of the candidate frame on the original image to the coordinates on the downsampled feature layer. The other time is when the feature map corresponding to the candidate box is divided into a grid of fixed size. Both quantization operations are rounded, so the position of the candidate box cannot be accurately expressed. Mask R-CNN proposes the ROI align method, which no longer performs rounding operations, but retains the floating point coordinates of the corresponding candidate boxes on the feature layer. It adopts the bilinear interpolation method to determine the pixel value in the grid to obtain a fixed-scale feature map. The pixel value is generated with bilinear interpolation from the four nearest pixels on the feature map of the candidate region. After obtaining the pixel value for the sampling point, the maximum pooling operation is performed on each subregion to obtain the feature map. The ROI align algorithm avoids the position error caused by the two quantization operations in ROI pooling without adding new parameters, which is beneficial to the refined positioning of dense targets in the creation of virtual reality digital media art.

### 3.5. Soft-NMS Algorithm

In target detection, the NMS algorithm is usually used as a post-processing step to delete redundant detections and retain the detection frame with the highest target score, and the NMS algorithm contains the following steps. First, coordinate information and category score probability value of all candidate boxes are selected under one of the categories, the candidate boxes are sorted in descending order with confidence, and the sequence number of the candidate box is obtained with the highest confidence. Second, all remaining candidate boxes are traversed and the IOU value between them and the candidate box is calculated with the highest confidence. IOU represents the ratio of the overlapping area of the two candidate frames to the combined area, which reflects the overlap between two candidate frames. The larger value, the higher degree of overlap. If the IOU value is greater than threshold, the candidate box is discarded. Third, the candidate frame with the highest confidence in the remaining candidate frames is selected, then other candidate frames and their IOU values are judged, and then the second candidate frame is retained. Fourth, the above process is iterated repeatedly, the candidate boxes are rough screened, and a certain number of candidate boxes are retained until all the candidate boxes meet the IOU threshold and the confidence score threshold, and the processing methods for other categories of candidate boxes are the same. NMS is calculated as follows:

(6) $$\begin{array}{c} s_{i}=\left\{\begin{array}{cc} s_{i}, & \text{IOU}<T,\\ 0, & \text{IOU}\geq T, \end{array}\right. \end{array}$$

where *s* is score and *T* is threshold.

The article "Application of Artificial Intelligence within Virtual Reality for Production of Digital Media Art" was published in 2022. Journal: Comput Intell Neurosci.

NMS algorithm is simple, fast, and has excellent performance, but NMS sets a hard threshold, and the selection of this threshold will directly affect the quality of the screening results. In the densely distributed area of targets, the distances between different targets are very close, so their bounding rectangles inevitably have overlapping areas. If the IOU threshold set by the NMS algorithm is too small, many suggestion boxes containing detection objects will be deleted by mistake, increasing the missed detection rate. On the contrary, if the IOU threshold set by the NMS algorithm is too large, the same detection target will be reserved for multiple proposal boxes, which will reduce the average detection accuracy. Therefore, the NMS algorithm is too absolute, and it is difficult to accurately retain the correct candidate boxes in different situations. To improve detection accuracy, this work adopts the soft-NMS algorithm for post-processing.

(7) $$\begin{array}{c} s_{i}=\left\{\begin{array}{cc} s_{i}, & IOU<T,\\ s_{i}\left(1-IOU\right), & IOU\geq T, \end{array}\right. \end{array}$$

where *s* is score and *T* is threshold.

The difference between the soft-NMS algorithm and the NMS algorithm is that it does not directly delete the candidate boxes whose IOU is higher than a given threshold, but attenuates their confidence, so that the proposed boxes of adjacent targets will not be missed. The larger IOU for two candidate boxes, the greater attenuation degree, because the greater the overlap rate, the more likely it is the proposed box of the same detection target. If the IOU value of the two candidate boxes is very small, the confidence score is not affected. The soft-NMS algorithm has a simple idea, does not increase the amount of new parameters, and does not increase the additional computational cost.

The article "Application of Artificial Intelligence within Virtual Reality for Production of Digital Media Art" was published in 2022. Journal: Comput Intell Neurosci.

## 4. Experiment and Discussion

### 4.1. Dataset and Environment

This work uses images collected from virtual reality digital media art creations as a dataset, including 90,837 training images and 30,871 test images, and it contains 103 types of targets. The experimental environment of this work is illustrated in Table 2.

The training process uses stochastic gradient descent, based on experience, the initial learning rate is 0.0001, and training iterations are 200 epochs. This work uses mAP and accuracy as evaluation indicators for target detection, and the calculation method is as follows:

(8) $$\begin{array}{c} \text{mAP}=\frac{1}{N}\sum_{i=1}^{N}AP_{i},\\ \text{Accuracy}=\frac{\left(TP+TN\right)}{\left(TP+TN+FP+FN\right)}. \end{array}$$

### 4.2. AODNET Training Loss

In the target detection task with deep learning, network training is necessary. This work evaluates the training process for AODNET and shows training loss, as demonstrated in Figure 3.

As the training iteration grows, the loss gradually decreases and finally stabilizes at around 0.5, at which point the network has converged.

### 4.3. Comparison with Other Detection Methods

To effectively prove the reliability of AODNET, it is compared with other detection methods, such as faster R-CNN, YOLO, and SSD. The comparison results of mAP and accuracy are demonstrated in Table 3.

Compared with other detection methods listed in the table, AODNET achieves the highest mAP and accuracy, 90.3% and 93.6%. Compared with the SSD method, these two performance indicators are improved by 2.4% and 2.2%, respectively.

### 4.4. Analysis on Combination of Faster R-CNN and ResNet

AODNET combines faster R-CNN and ResNet networks. To verify the superiority of this combined strategy, mAP and accuracy are compared between uncombined and combined. To ensure the reliability of the experiment, the rest of the network parameter settings remain unchanged, and the results are demonstrated in Figure 4.

As can be seen from the data comparison in the figure, when faster R-CNN and ResNet are combined, the mAP is increased by 4.4% and the accuracy rate is increased by 2.8% compared with performance when they are not combined. This shows that the combination of faster R-CNN and ResNet can mine deep features more effectively.

### 4.5. Analysis on Candidate Box Optimization

AODNET utilizes K-means++ for size optimization of candidate box. To verify the superiority of this method, it is compared with the original candidate frame selection strategy and the K-means optimization strategy. The mAP and accuracy corresponding to the three methods are demonstrated in Figure 5.

The article "Application of Artificial Intelligence within Virtual Reality for Production of Digital Media Art" was published in 2022. Journal: Comput Intell Neurosci.

Compared with the original candidate box selection strategy, using the clustering algorithm for optimization can achieve a certain degree of performance improvement. However, the mAP and accuracy corresponding to the K-means++ algorithm are the highest. Compared with K-means optimization, index improvement of 2% and 1.3% is obtained.

### 4.6. Analysis on ROI Align

AODNET replaces the ROI pooling in the original faster R-CNN with ROI align. To verify the superiority of this replacement strategy, the performance of using ROI pooling and using ROI align is compared, respectively. The mAP and accuracy of the two are compared in Figure 6.

Compared with using ROI pooling, after using ROI align, the mAP and accuracy of AODNET are improved by 2.2% and 1.1%, respectively. This is mainly because ROI align reduces the error caused by two quantizations, thereby improving the robustness and discrimination of features.

### 4.7. Analysis on Soft-NMS

AODNET uses soft-NMS to process the detection frame. To verify its superiority compared with traditional NMS, this work compares the mAP and accuracy when using NMS and soft-NMS, respectively, as demonstrated in Figure 7.

As can be seen from the data comparison in the figure, when using soft-NMS, the mAP is increased by 1.6% and accuracy rate is increased by 0.7% compared with performance when using traditional NMS.

### 4.8. Analysis on Training Batch

In deep neural network training, the training batch is variable. To verify the impact of different batches on the detection performance, this work compares the mAP and accuracy rates corresponding to different batch sizes, as demonstrated in Table 4.

When batch changes, the mAP and accuracy of AODNET will also change dynamically, and the overall change shows a trend of rising first and then falling. When the batch size is set to 32, the highest mAP and accuracy can be obtained.

## 5. Conclusion

Industry and academics have paid increasing attention to virtual reality technology in recent years. Users can interact with virtual items using numerous interactive methods thanks to virtual reality technology, which generates realistic visuals, sounds, and other sensory experiences using computer technology. Artificial intelligence has advanced rapidly in tandem with computer technology. As digital media art continues to evolve, virtual reality and artificial intelligence have become the primary tools for creating new works of art. Aiming at particularity for object detection in digital media art creation of VR, this work proposes an art object detection algorithm based on residual network and clustering idea. First of all, it uses ResNet50 as the feature extraction network, which deepens the network depth and improves the model feature extraction ability. Second, it uses the K-means++ algorithm to perform clustering statistics on the size of the real annotated boxes in the dataset to obtain appropriate hyperparameters for preset candidate boxes, which enhances the tolerance of the algorithm to the target size. Third, it replaces the ROI pooling algorithm with ROI align to eliminate the error caused by the quantization operation on the characteristics of the candidate region. Fourth, to reduce missed detection rate of overlapping targets, soft-NMS algorithm is used instead of the NMS algorithm to post-process the candidate boxes. Finally, this work conducts extensive experiments to verify the superiority of AODNET for object detection in virtual reality digital media art creation.

The article "Application of Artificial Intelligence within Virtual Reality for Production of Digital Media Art" was published in 2022. Journal: Comput Intell Neurosci.

## Figures and Tables

**Figure 1:** Residual unit.

**Figure 2:** Combination of ResNet and faster R-CNN.

**Figure 3:** AODNET training loss.

**Figure 4:** Analysis on combination of Faster R-CNN and ResNet.

**Figure 5:** Analysis on candidate box optimization.

**Figure 6:** Analysis on ROI align.

**Figure 7:** Analysis on soft-NMS.

**Table 1:** ResNet50 structure.

Layer	Parameter
Conv 1	7 × 7, 3 × 3, Maxpooling
Conv 2	[1× 1, 3 × 3, 1 × 1] × 3
Conv 3	[1 × 1, 3 × 3, 1 × 1] × 4
Conv 4	[1 × 1, 3 × 3, 1 × 1] × 6
Conv 5	[1 × 1, 3 × 3, 1 × 1] × 3
Average pooling	14 × 14
FC	1000
Softmax	1000

**Table 2:** Experimental environment details.

Name	Parameter
GPU	GTX 1080Ti 16 GB
CPU	Intel Core i5-9300H
System	Ubuntu 18.04
Language	Python
Framework	PyTorch

**Table 3:** Comparison with other detection methods.

Method	mAP	Accuracy
Faster R-CNN	83.8	86.4
YOLO	86.1	89.5
SSD	87.9	91.4
AONET	90.3	93.6

**Table 4:** Analysis on training batch.

Batch size	8	16	32	64	128
mAP	85.3	88.9	90.3	89.5	87.5
Accuracy	90.9	92.6	93.6	93.1	91.2

## Data Availability

The datasets used during this study are available from the corresponding author on reasonable request.
